# Expression and Clinical Significance of Serum Krüppel-Like Factor 7 (KLF7) in NSCLC Patients

**DOI:** 10.1155/2022/9270789

**Published:** 2022-07-27

**Authors:** Huigai Song, Jingjing Sun, Zhiming Xu, Xinru Liu, Na Liu

**Affiliations:** ^1^Pathology Department, Hebei Chest Hospital, Shijiazhuang, Hebei 050000, China; ^2^Department of Immunization Planning, Chengde Center for Disease Control and Prevention, Chengde, Hebei 067000, China

## Abstract

Nonsmall cell lung cancer (NSCLC) is a serious threat to the life and health of patients with high incidence rate and mortality. The present research was to assess the relationship between the serum Krüppel-like factor 7 (KLF7) level and the recurrence and metastasis of NSCLC patients. 150 patients with NSCLC treated by thoracoscopic radical resection of lung cancer in our hospital from January 2016 to February 2017 were selected. As the control group, 148 healthy people who went to the hospital for physical examination in the same period were screened. The expression levels of serum KLF7 in the observation group and the control group were compared and analyzed. According to the level of KLF7 expression, the patients in the observation group were divided into KLF7 high expression group (≥258.6 ng/L, *n* =75) and KLF7 low expression group (<258.6 ng/L, *n* =75). The 3-year recurrence and metastasis rate of patients in each group was compared and analyzed. It was found the concentration of serum KLF7 in peripheral blood of NSCLC (2.25 ± 0.65) ng/ml was significantly higher than that in healthy population (1.42 ± 0.38) ng/ml (*P* < 0.05). The expression level of serum KLF7 was not related to gender, age, smoking history, and tumor diameter of NSCLC patients (*P* > 0.05), but related to the degree of differentiation and TNM stage of NSCLC patients (*P* < 0.05). Univariate analysis showed that the degree of differentiation, TNM stage, and KLF7 were significantly correlated with 3-year recurrence and metastasis of NSCLC patients (*P* < 0.05). Cox regression analysis showed that low degree of differentiation, TNM stage IIIa, and KLF7 were independent risk factors for recurrence and metastasis in NSCLC patients in 3 years (*P* < 0.05). Taken together, the expression level of serum KLF7 in patients with NSCLC is significantly increased, which is an independent risk factor for recurrence and metastasis in 3 years, and is worthy of clinical application.

## 1. Introduction

Lung cancer is the leading cause of death worldwide, with high incidence rate and mortality [1–5]. Nonsmall cell lung cancer (NSCLC) refers to all epithelial cell lung cancer except small cell lung cancer. At present, it is mainly treated by surgical resection, radiotherapy, and chemotherapy, with good clinical efficacy. However, some patients can still have distant metastasis and recurrence, which seriously affects the prognosis [6–8]; therefore, timely assessment of the risk of recurrence and metastasis after treatment can formulate a reasonable clinical treatment plan in advance, so as to significantly improve the prognosis of patients [9, 10]. Therefore, it is particularly important to study the biological characteristics of lung cancer and find the method of early detection of lung cancer to improve the cure rate and prognosis of lung cancer.

Krüppel-like factor 7 (KLF7) is a member of specificity protein/Krüppel-like factor (SP/KLF) family. It is widely expressed at low and medium levels in adult tissues. Functional studies show that KLF7 plays an important role in the development of the nervous system and adipogenesis and is a gene related to many diseases [11–13]. Recent studies have shown that KLF7 is also involved in many new biological processes, such as sciatic nerve regeneration [14, 15], mediating tissue inflammatory response [16], participating in cancer radiotherapy [17] and chemotherapy rehabilitation, regulating oxidative phosphorylation pathway [18], and so on. Furthermore, it has been reported that KLF7 can enhance the ability of tumor migration and invasion, which is related to tumor recurrence and metastasis [19, 20], whereas there are few studies on its expression in the serum of patients with NSCLC. Based on this, this study explored the relationship between the expression level of serum KLF7 and the recurrence and metastasis of NSCLC patients, in order to provide reference for predicting the recurrence and metastasis of NSCLC in advance. The report is as follows.

## 2. Clinical Data

150 patients with NSCLC treated by thoracoscopic radical resection of lung cancer in our hospital from January 2016 to February 2017 were selected as the observation group, including 100 males and 50 females; the age ranged from 47 to 74 years, with an average of (56.25 ± 8.42) years; 72 cases had tumor diameter ≥4 cm and 78 cases had tumor diameter<4 cm; 60 cases were poorly differentiated and 90 cases were moderately well differentiated; TNM stages were stage I in 50 cases, stage II in 35 cases, and stage IIIa in 65 cases. The informed consent form was signed with the patients before the clinical study and approved by the ethics committee of the hospital. The serum of the healthy control group was taken from 148 healthy subjects in the same period in the physical examination center of our hospital, including 101 males and 47 females,; The age ranged from 46 to 74 years, with an average of (56.32 ± 8.25) years. There was no significant difference in gender and age between pathological group and healthy control group. Inclusion criteria: (1) no specific treatment for lung cancer, including surgery, radiotherapy, chemotherapy, targeted drug therapy, and biotherapy, was received before admission; (2) patients with lung cancer confirmed by fiberscope biopsy, percutaneous needle aspiration biopsy, or postoperative pathology were classified according to the classification standard of lung cancer tissue issued by the World Health Organization (WHO) in 2015, and the lung cancer was staged according to the 8^th^ edition of lung cancer primary tumor lymph node metastasis (TNM) staging system issued by the International Anti Cancer Alliance in 2017.

## 3. Methods

The fasting peripheral blood of NSCLC patients and healthy controls was collected with Ethylenediamine tetraacetic acid (EDTA) anticoagulant tube, stored in 4°C refrigerator for temporary storage, and sent to the laboratory within 24 h. After low-temperature and high-speed centrifugation, the serum was sub-packed and tested in -80°C refrigerator. The double antibody sandwich enzyme-linked immunosorbent assay (ELISA) was used to detect KLF7, which was operated in strict accordance with the instructions of ELISA Kit (R&D, USA).

The standard curve was drawn through the solution of standard KLF7 protein concentration and its OD_450_, and the serum OD_450_ of healthy people and lung cancer patients was detected, respectively, so as to calculate the serum KLF7 concentration, and the serum KLF7 levels of healthy people and lung cancer patients were compared, respectively; in patients with NSCLC, they were compared according to their age, gender, smoking history, tumor size, pathological type, degree of tumor differentiation, lymph node metastasis, and clinical stage.

## 4. Observation Index

All patients were treated with thoracoscopic radical resection of lung cancer. They were followed up for 3 years by outpatient and telephone. The starting time of follow-up was the recurrence and metastasis of CT examination or the last follow-up was the end of follow-up. All patients were followed up successfully. (1) The expression levels of serum KLF7 in the observation group and the control group were compared and analyzed. (2) To analyze the relationship between the expression level of serum KLF7 and the clinicopathological features of NSCLC patients. (3) According to the level of KLF7 expression in the observation group (taking the average value of its expression level as the dividing line), they were divided into KLF7 high expression group (≥258.6 ng/L, *n* =75) and KLF7 low expression group (<258.6 ng/L, *n* =75). The 3-year recurrence and metastasis rate of patients in NSCLC was compared and analyzed. (4) To analyze the influencing factors of 3-year recurrence and metastasis in patients with NSCLC (Figure 1).

## 5. Results

### 5.1. Comparison of Serum KLF7 Concentration in Peripheral Blood

The serum KLF7 concentration in peripheral blood of NSCLC (2.25 ± 0.65) ng/ml was markedly higher than that in healthy population (1.42 ± 0.38) ng/ml, and the divergence was statistically prominently (*P* < 0.05).

### 5.2. Single Factor Analysis of Serum KLF7 in Patients with NSCLC

The expression level of serum KLF7 was not related to gender, age, smoking history, and tumor diameter of NSCLC patients (*P* > 0.05) but significantly related to the degree of differentiation and TNM stage of NSCLC patients (*P* < 0.05) (see Table 1).

### 5.3. Analysis of 3-Year Recurrence and Metastasis in Patients with NSCLC

Univariate analysis showed that the degree of differentiation, TNM stage, and KLF7 were significantly correlated with 3-year recurrence and metastasis of NSCLC patients (*P* < 0.05). TNM stage IIIa and KLF7 were independent risk factors for recurrence and metastasis of NSCLC patients in 3 years was Cox regression analysis clarified (*P* < 0.05) (see Tables 2 and 3).

## 6. Discussion

With the change of living environment and air quality, the number of lung cancer patients has a high trend. According to relevant data, the number of new lung cancer patients worldwide is more than 1.8 million every year, while China's lung cancer data in 2015 shows 733000 new cases and more than 610000 deaths. Lung cancer is the most common malignant tumor in the clinic [21–23], and the most common pathological type is NSCLC, which mainly includes squamous cell carcinoma (SCC), adenocarcinoma (LAC), and large cell carcinoma (LCC) [24–26]. With the development of precision medicine, chemotherapy, radiotherapy, targeted therapy, and immunotherapy have prolonged the survival of some patients with advanced lung cancer, but the 5-year survival rate is still less than 21% [27–30]. Therefore, it is of great clinical significance to find a simple and easy to operate prognostic evaluation index. So far, the immune function has attracted attention of patients with lung cancer. Studies have shown that the occurrence, development, metastasis, and recurrence of malignant tumors are related to the defects of immune function [31–33]. Patients with lung cancer have a certain degree of abnormal immune function [34, 35]. In recent years, with the rise and development of molecular biology, tumor drug therapy has shown a diversified trend. Among them, molecular targeted drugs have become a hot spot in the clinical treatment of nonsmall cell lung cancer because of their strong pertinence and high safety. Moreover, the continuous development of multidisciplinary comprehensive treatment methods such as molecular targeted therapy and immunotherapy has provided a new direction for the clinical treatment of lung cancer and enriched the means of lung cancer treatment [36–38]. With the in-depth study of the immune tolerance mechanism of lung cancer, the interaction of KLF7 in the occurrence and development of lung cancer has attracted more and more attention of scholars at home and abroad.

The research on KLF7 in the serum of cancer patients is not uncommon. The research shows that the research on KLF7 in the serum of cancer patients is not uncommon. At present, a research has found that the serum KLF7 level of breast cancer patients is higher than that of healthy people [39]; furthermore, a study has found that the level of serum KLF7 has diagnostic significance for gastrointestinal cancer [11]. The research on the correlation between KLF7 and NSCLC is mainly concentrated in lung cancer tissues and cells [40], and its research in the serum of lung cancer patients is relatively few. The research results mostly suggest that KLF7 has a positive correlation with the malignant degree of NSCLC, which is consistent with the findings of this study. The mechanism of KLF7 promoting tumor may be related to KLF7 promoting the invasion of tumor cells into microvessels and promoting the formation of neovascularization.

At present, the study has found that the expression of serum KLF7 in patients with lung cancer is significantly higher than that in healthy people [41], suggesting that KLF7 is expected to become a new tumor marker. In patients with lung cancer, the expression level of serum KLF7 had nothing to do with the gender, age, smoking history, and tumor diameter of patients with NSCLC. However, the level of serum KLF7 in patients with low differentiation was higher than that in patients with high differentiation. The concentration of serum KLF7 in patients with clinical stage IIIa was significantly higher than that in patients with stage I~II, suggesting that KLF7 may have a positive correlation with the degree of malignancy of patients and may have a certain value for the prognosis of lung cancer. The 3-year recurrence and metastasis rate of KLF7 high expression group was significantly higher than that of KLF7 low expression group, and KLF7 was an independent risk factor for recurrence and metastasis 3 years after operation. The results showed that the expression level of KLF7 increased and participated in the recurrence and metastasis of NSCLC. The study also found that TNM stage IIIa was an independent risk factor for 3-year recurrence and metastasis of NSCLC patients. It is considered that the cancer at this stage may have spread outside the lung and it is difficult to completely eliminate the cancer by surgical treatment. In conclusion, the expression level of serum KLF7 in patients with NSCLC is significantly increased, which is an independent risk factor for recurrence and metastasis in 3 years. It has a high efficiency in predicting recurrence and metastasis in 3 years after operation, which is worthy of clinical application. However, this study is a single-center study. Only NSCLC patients treated with thoracoscopic radical resection of lung cancer and NSCLC patients not treated with radiotherapy and chemotherapy may have selection bias in the results. At the same time, the follow-up time is short, and further research is needed in the follow-up.

The advantages of molecular targeted therapy are targeting safety and convenience. Compared with traditional chemotherapy, molecular targeted therapy can reduce the pain of patients' clinical treatment as much as possible [42]. At present, targeted therapy has gradually completed the development goal of individualized and accurate treatment. At the same time, it is committed to carrying out comprehensive treatment with multiple disciplines. Its application in clinical treatment is also gradually popularized, avoiding the pain of patients caused by chemotherapy to the greatest extent. The emergence of molecular targeted therapy has opened up a new field for the clinical treatment of lung cancer. It has the advantages comparable to traditional chemotherapy and is an important link in the clinical standard treatment of modern medical lung cancer. How to maximize the benefits of molecular targeted therapy in tumor treatment and give the most effective “one-to-one” clinical treatment scheme to individual patients has become a hot topic in medical tumor treatment. With the development of molecular targeted therapy, there are still many problems to be solved. In a word, with the continuous exploration of molecular targeted therapy, the mechanism of molecular targeted therapy will be more and more clear. How to formulate a targeted plan for the treatment based on the actual situation and tolerance of patients and how to use molecular targeted therapy to prolong the survival time of patients are a subject of continuous medical research.

## Figures and Tables

**Figure 1:** Summary images.

**Table 1:** Single factor analysis of serum KLF7 in patients with NSCLC (^−^*x* ± *s*).

Characteristic	Cases (*n*)	KLF7	*t*	*P*
Gender			0.145	0.885
Male	100	2.15 ± 0.32		
Female	50	2.13 ± 0.52		
Age			0.870	0.386
≥60	78	2.25 ± 0.42		
<60	72	2.32 ± 0.56		
Smoking history			0.443	0.658
Have	80	2.12 ± 0.23		
No have	70	2.14 ± 0.32		
Tumor diameter			0.698	0.486
≥4 cm	68	2.32 ± 0.54		
<4 cm	82	2.26 ± 0.51		
Degree of differentiation			5.134	0.001
Low differentiation	55	2.41 ± 0.41		
Medium and high differentiation	95	2.15 ± 0.21		
TNM staging			5.274	0.001
Phase I~II	85	2.04 ± 0.42		
Phase IIIa	65	2.38 ± 0.35		

Note: *P* value represents the difference with statistical significance.

**Table 2:** Univariate analysis of 3-year recurrence and metastasis rate in patients with NSCLC (*n*, %).

Characteristic	3-year recurrence and metastasis rate (*n*, %)	*X* ^2^	*P*
Gender		0.240	0.624
Male	68 (68)		
Female	32 (64)		
Age		0.366	0.545
≥60	45 (57.69)		
<60	38 (52.77)		
Smoking history		2.228	0.135
Have	56 (70)		
No have	36 (51.43)		
Tumor diameter		2.636	0.104
≥4 cm	50 (73.53)		
<4 cm	50 (60.97)		
Degree of differentiation		6.981	0.008
Low differentiation	45 (81.82)		
Medium and high differentiation	58 (60.05)		
TNM staging		6.803	0.009
Phase I~II	48 (56.47)		
Phase IIIa	50 (76.92)		
KLF7		8.466	0.003
≥258.6 ng/L	62 (82.67)		
<258.6 ng/L	45 (61.33)		

Note: *P* value represents the difference with statistical significance.

**Table 3:** Cox regression analysis of 3-year recurrence and metastasis rate in patients with NSCLC.

Influence factor	*β*	SE	Wald *X*^2^	*P*	HR (95% CI)
The degree of differentiation is low	0.396	0.207	3.856	0.043	1.472 (1.012~2.225)
TNM stage is IIIa stage	0.368	0.202	3.821	0.048	1.485 (1.325~2.684)
KLF7	0.725	0.206	7.815	0.004	2.084 (1.396~3.105)

Note: *P* value represents the difference with statistical significance.

## Data Availability

The datasets used and analyzed during the current study are available from the corresponding author upon reasonable request.
